# Antimicrobial Potential of *Pithecellobium dulce* Seed Extract against Pathogenic Bacteria: In Silico and In Vitro Evaluation

**DOI:** 10.1155/2023/2848198

**Published:** 2023-02-04

**Authors:** Abdu Aldarhami, Abdulrahman S. Bazaid, Abdullah S. Alhamed, Adel F. Alghaith, Syed Rizwan Ahamad, Yasseen A. Alassmrry, Talal Alharazi, Mejdi Snoussi, Husam Qanash, Abdulwahab Alamri, Riadh Badraoui, Adel Kadri, Naif K. Binsaleh, Mousa Alreshidi

**Affiliations:** ^1^Department of Medical Microbiology, Qunfudah Faculty of Medicine, Umm Al-Qura University, Al-Qunfudah 21961, Saudi Arabia; ^2^Department of Medical Laboratory Science, College of Applied Medical Sciences, University of Ha'il, Hail 55476, Saudi Arabia; ^3^Department of Pharmacology & Toxicology, College of Pharmacy, King Saud University, Riyadh 11451, Saudi Arabia; ^4^Department of Pharmaceutics, College of Pharmacy, King Saud University, Riyadh 11451, Saudi Arabia; ^5^Central laboratory, Department of Pharmaceutical Chemistry, College of Pharmacy, King Saud University, Riyadh 11451, Saudi Arabia; ^6^Department of Clinical Microbiology and Immunology, Faculty of Medicine and Health Sciences, Taiz University, Yemen; ^7^Department of Biology, College of Science, University of Ha'il, Hail 55476, Saudi Arabia; ^8^Laboratory of Genetics, Biodiversity and Valorization of Bio-Resources (LR11ES41), University of Monastir, Higher Institute of Biotechnology of Monastir, Avenue Tahar Haddad, BP74, Monastir 5000, Tunisia; ^9^Molecular Diagnostics and Personalized Therapeutics Unit, University of Ha'il, Hail 55476, Saudi Arabia; ^10^Department of Pharmacology and Toxicology, College of Pharmacy, University of Ha'il, Hail 55211, Saudi Arabia; ^11^Section of Histology-Cytology, Medicine Faculty of Tunis, University of Tunis El Manar, La Rabta, Tunis 1007, Tunisia; ^12^College of Science and Arts in Baljurashi, Al Baha University, Al Baha 65515, Saudi Arabia; ^13^Faculty of Science of Sfax, Department of Chemistry, University of Sfax, B.P. 1171, Sfax 3000, Tunisia

## Abstract

Clinical multi-drug-resistant bacteria continue to be a serious health problem. Plant-derived molecules are an important source of bioactive compounds to counteract these pathogenic bacteria. In this paper, we studied the chemical composition of the methanol (80%) extract from *Pithecellobium dulce* seed (Hail, Saudi Arabia) and its ability to inhibit the growth of clinically relevant multi-drug-resistant bacteria. Molecular docking analysis was performed to predict the best compounds with low binding energy and high affinity to interact with two *Staphylococcus aureus* receptors. Data showed that *P. dulce* extract is a rich source of D-turanose (55.82%), hexadecanoic acid (11.56%), indole-1-acetic acid (11.42%), inositol (5.78%), and octadecanoic acid (4.36%). The obtained extract showed antibacterial activity towards tested clinical bacterial strains with MIC values ranging from 233 mg/mL for *Acinetobacter baumannii* to 300 mg/mL for *S. aureus* and *Escherichia coli*. Turanose interaction has resulted in -7.4 and -6.6 kcal/mol for 1JIJ and 2XCT macromolecules, while inositol showed energy values (−7.2 and −5.4 kcal/mol) for the same receptors. Multiple identified compounds showed desirable bioavailability properties indicating its great potential therapeutic use in human. Overall, current investigation highlights the possible use of *P. dulce* extract as a valuable source for drug development against pathogenic drug-resistant bacteria.

## 1. Introduction

Owing to the extensive use of antibiotics, antimicrobial resistance (AMR) has become a major heath concern worldwide [1]. Accordingly, the ongoing emergence of resistant isolates towards multiple currently utilised antibiotic drugs has limited its effectiveness to treat several bacterial infections [1]. Bacterial isolates that are resistant to two classes of antibiotics are defined as multi-drug-resistant (MDR) bacteria, which carries the highest rate of mortality compared to infections caused by non-MDR bacteria [2]. Gram-negative bacteria, including *Escherichia coli*, have overtaken MDR infections due to the limited availability of effective antibiotic drugs against this group of bacteria [3]. In Saudi Arabia, 29%, 65%, and 11% of isolated *E. coli*, *Klebsiella pneumoniae*, and *Acinetobacter baumannii* were identified as extended spectrum beta-lactamase- (ESBL-) producing isolates, respectively [4]. These facts about the widespread of AMR, ineffective antibiotics drugs, and the low rate of discovery for new antibiotics are clearly posing one of the serious and greatest threats to the public healthcare worldwide [5]. Thus, actions to tackle/control the spread of AMR, including the discovery and characterisation of new antimicrobial compounds, are urgently required [6].

Before the 21st century, about 11% (252) of the WHO's basic and necessary medications have entirely been made from flowering plants [7]. Currently, it was claimed that between 35,000 and 70,000 plant species have been evaluated for medicinal potential [7]. Various natural products (NPs) are currently and widely used based on laboratory research as a healing component for numerous deadly diseases, severe cancers, for instance [8, 9]. Additionally, endless of blockbuster medications that are clinically used today were originated from plants by different means [6]. Namely, plant-derived medicines have a long history of therapeutic usage in human with desirable level of safety (patient friendly) and potent activity towards pathogens, which has a role in the improved human health [6]. Given information would highlight the importance of plants as valuable source for the discovery of potentially novel antibacterial compounds with limited toxicity and desirable bioavailability and pharmacodynamics features for the treatment of infections caused by drug-resistant bacteria.

In the last decade, the field of plant-derived medicine has witnessed more interest by researchers globally with high demand for the extraction of therapeutic compounds to treat infectious and noninfectious illness [10]. In addition, about 80% of used traditional medicines in developing country are plant-derived, including *Pithecellobium* [11]. There are various species of *Pithecellobium* that are found in the tropics, primarily in Asia and North America, which belong to the Leguminosae family [12]. *Pithecellobium dulce* is the most well-known species that is commonly referred to as Jungle Jalebi or Manila, which is an evergreen, small- to medium-sized tree of 18 m in height [12]. Several remedies are associated with *Pithecellobium dulce*, including a folk that is used to treat toothaches, earaches, ulcers, leprosy, and peptic ulcers [13]. In addition, *Pithecellobium dulce* is also used in another folk medications as an anodyne, emollient, and larvicide [13]. Moreover, skin of the stem of *Pithecellobium dulce* is traditionally utilised to treat dysentery [14]. Leaves, roots, and seeds of this plant species are claimed to treat intestinal disorders and ulcers while leaves were claimed to relieve pain associated with venereal sores [14, 15]. Furthermore, multiple reports have claimed an anti-inflammatory effect caused by the extract of *Pithecellobium dulce* [12].

Nevertheless, limited investigations were conducted on the antimicrobial activity of *Pithecellobium dulce*. Root extract of *Pithecellobium dulce* has revealed promising antibacterial activity against *Staphylococcus aureus*, *Klebsiella pneumonia*, and *Enterobacter aerogenes* [16], while seed extract has inhibited the growth of *E. coli* and *Pseudomonas aeruginosa* [17]. Several unique and interesting metabolites that have been isolated from different parts of this plant were screened for bioactivity [18]. However, there are several aspects of this plant still unexplored including the interaction between compounds of this extract and sensitive bacterial targets, despite the impressive literature in relation with chemical, pharmacological, and clinical investigations. Thus, the aim of this project was to investigate phytochemicals, antimicrobial activity against pathogenic bacteria, and molecular docking of *Pithecellobium dulce* seed extract.

## 2. Materials and Methods

### 2.1. Extraction Process

Seeds were collected from *Pithecellobium dulce* tree (Hail region, Saudi Arabia) and washed with sterile distilled water. Around 400 grams of *P. dulce* seed was ground to a coarse powder using an electrical grinding mill and extracted by cold maceration in 80% methanol (Sigma-Aldrich, MO, USA) at room temperature [19]. It was then left standing for 3-4 days with an occasional shaking to produce the crude extract. Later, the crude extract was filtered using Whatman® qualitative filter paper (grade 1, 45 mm) (Wagtech International Ltd., England). Then, filtered product was concentrated using a rotary vacuum evaporator (Buchi Rotavap) at reduced pressure (45 rpm) and temperature (40°C). After drying, around 6 grams of the powder extract was produced and stored at 4°C.

### 2.2. GC-MS Analysis

The GC-MS analysis was performed using as Perkin Elmer model Clarus 600 T combined with single quadrupole mass spectrometer [20]. Briefly, elite 5-MS column (30 m × 0.25 mm × 0.25 *μ*m film thickness) with high-purity helium gas carrier at a flow rate of 1 mL/min was utilised in this experiment. The injector temperature of the injector was set at 280°C that was equipped with a splitless injector at ratio 20 : 1. The temperature was set initially to 40°C (held for 1 min), then further increased to 150°C at 10°C per min, and then increased further to 300°C at 10°C per min (held for 3 min). Temperatures of the MS ion source and inlet line were 200°C and 220°C, respectively. The range of scanning for mass was set between 40 and 618 m/z, and the electron energy for ionization was 70 eV. The filament of mass starts after 7 min to elute peaks from the solvent. Obtained peaks were identified using the National Institute of Standard and Technology (NIST) library (2005 software) and Wiley library (2006).

### 2.3. Derivatization of Plant Extract

Around 300 *μ*L of the plant extract was taken and dried completely using nitrogen air. Then, methoxymation was carried out at room temperature by adding 100 *μ*L of methoxyamine hydrochloride in pyridine solution (20 mg/mL). The mixture was vortexed for 10 min and was then left for 16 hours at room temperature. The methoxymated sample underwent a derivatization reaction by using 100 *μ*L of BSTFA/TMCS (N,O-bis(trimethylsilyl)trifluoroacetamide with trimethylchlorosilane) (99/1, *v*/*v*) and vortexed for 10 minutes. The solution was then maintained for 2 hours at 50°C prior the completion of derivatizing reaction. Later, 1 *μ*L of the derivatized sample was injected into the system in a split mode (split ratio 1 : 20).

### 2.4. Antibacterial Activity of Plant Extract

Different clinical bacterial isolates, including *Staphylococcus aureus*, *Escherichia coli*, and drug-resistant *Acinetobacter baumannii*, were collected from King Khalid Hospital in Hail for testing the activity of plant extract. The antimicrobial activity of the extract was determined using the agar well diffusion method and broth microdilution method [21]. Overnight bacterial suspension was diluted 1 : 100 and was spread over the entire Muller-Hinton agar (MHA) using sterile cotton swab. Then, a hole with a diameter of 6 mm was made with a sterile cork-borer, and 100 *μ*L of the extract (80% *v*/*v*) was inoculated into the well. Ceftriaxone (30) antibiotic disc was used as positive control. MHA plates were incubated for overnight, and zone of inhibition was measured in millimetre (mm). For broth microdilution method, 100 *μ*L of bacterial suspension at optical density (OD of 0.08) for each tested bacterial isolate was made and transferred then to designated wells using 96-well plate. Multiple concentrations (100-1000 mg/mL) of plant extract were made by dissolving the extract in a sterile distilled water and 5% dimethyl sulfoxide (DMSO). Then, the prepared concentrations were added to the different wells that were inoculated with bacterial isolates. Bacterial culture and sterile broth were included as positive and negative controls, respectively. Minimum inhibitory concentration (MIC) was determined by observing the lowest concentration that visually inhibited the bacterial growth (clear well) after 24 hours of incubation at 37°C. 10 *μ*L of well that showed no bacterial growth was transferred to a sterile Mueller-Hinton Agar (MHA) and further incubated for 24 hours at 37°C. Minimum bactericidal concentration (MBC) was defined as the lowest concentration exhibited absent of any bacterial colonies.

### 2.5. In Silico Simulation and Molecular Interactions

The antimicrobial activity of the identified extract components was further confirmed by in silico molecular docking and interaction assay against *S. aureus*. *S. aureus* was selected for this experiment as it was presented with a slightly larger inhibitory zone against the extract in comparison with tested Gram-negative bacteria. In this context, two receptors from *S. aureus* (1jij and 2xct) have been targeted: TyrRS and gyrase, for tyrosyl-tRNA synthetase and type IIa topoisomerase, respectively. These receptors were selected because they are commonly associated with the microbial function, particularly with *S. aureus* infections [22, 23]. The tridimensional structure of the targeted receptors was obtained by using RCSB protein data bank. ChemDraw was applied to draw the chemical structures of the identified compound, which then have been saved in PDB database [24]. The targeted receptors were preprocessed before docking analysis, based on the CHARMM force field; then, binding affinity and hydrogen bonding were calculated MGL tools and Vina® packages [25]. Compounds exhibiting best binding energy and high abundance in the extract were selected for 2D diagram of interactions with two *S. aureus* receptors.

### 2.6. ADMET Prediction

Prediction of physicochemical, pharmacokinetic, and drug-likeness properties of major compounds was investigated by SwissADME web-based tool (http://www.swissadme.ch/) [26].

## 3. Results and Discussion

### 3.1. Phytochemical of Pithecellobium dulce Seed Extract

Phytochemical profile of Pithecellobium dulce seed extract was determined when conducting a GC-MS that showed the presence of multiple compounds with molecular weight (MW) ranged from 90 to 353 g/mol, including the potentially active compound/s (Table 1). The extract is made of a range of compounds with various percentages of availability counting, D-turanose (55.8%), inositol derivatives (6.5%), hexadecanoic acid (12%), dihydroxyacetone (1.6%), D-gluco-hexodialdose (0.8%), 2-deoxy-galactopyranose (0.2%), ribitol (0.2%), D-mannose (0.2), and altronic acid (0.65%). Pithecellobium dulce seed contains high concentration of different sugars including D-turanose (3-O-*α*-D-glucopyranosyl-D-fructose). The majority of these sugars are well reported as plant metabolites, including Pithecellobium dulce, which have been linked to various activities, such as antioxidant, antitumor, and/or antibacterial activities [27]. Nevertheless, D-turanose revealed to be the most abundant component making more than half of the extract providing higher probability of being responsible for the tested activity. The availability of sugars (e.g., D-turanose) in high concentration is a well-reported mode of action by which bacterial growth is inhibited [28]. This is because the elevated osmotic pressure on bacterial cells resulted from the high level of sugar causing its burst and/or shrinkage leading to bacterial death [28]. For instance, antimicrobial activity of various tested honeys is more often linked with the high concentration of sugar [29]. In addition, D-turanose sugar has been revealed in certain type of honeys and Ziziphus spina-christi leaves that showed antibacterial activity [27]. Hence, it is highly expected that D-turanose sugar is the main responsible compound for the current antibacterial activity form the extract of *P. dulce* seed.

Nevertheless, organic saturated or unsaturated fatty acids, fatty acid esters (FAEs), and alcoholic compounds were detected in the GC-MS analysis of the tested extract (Table 1), which might possess antimicrobial properties. Data of this GC-MS spectra would concur with the previous investigation on plant leaves of *P. dulce* where multiple compounds including sugars, fatty acids, alkaloids, flavonoids, saponins, coumarin, tannins, anthocyanin, and triterpenoids were observed, and the antimicrobial activity was claimed for this mixture of compounds presented in the leave extract [13]. In addition, the analysis of Benth extract showed high concentration of saturated and unsaturated fatty acids that was linked with its antibacterial properties [30]. This is because fatty acids are well known for the ability to kill bacterial cells by either disruption their cell membranes or suppression the synthesis of fatty acids [21, 31]. For example, long chain fatty acids, including hexadecanoic and 9-octadecenoic acids (Table 1) that have been naturally occurring in various food products (e.g., olive oil, butter milk, and cheese) as well as in the *Pithecellobium dulce* seed, have been reported for the ability to inhibit the growth of *S. aureus* by interfering with enoyl-acyl carrier protein reductase (FabI), which has been an essential fatty acid synthesis enzyme [30, 32]. In addition, hexadecanoic acid has showed activity against MDR, including *S. aureus*, *K. pneumoniae*, and *P. aeruginosa* [33]. Hexadecanoic acid was observed on the extract of Andrographis paniculata leave, Albizia adianthifolia, and Pterocarpus angolensis that was reported as being the main compound behind the antimicrobial activity of these extracts towards Gram-negative (e.g., *E. coli* and *P. aeruginosa)* and Gram-positive (e.g., *S. aureus* and *Bacillus subtilis*) bacteria [34]. Furthermore, 9,12-octadecadienoic and hexadecanoic acid are two components that were predominant in the extract of Peperomia pellucida leaf that displayed activity against *E. coli*, *P. aeruginosa*, and *Vibrio cholerae* [35]. Therefore, the antimicrobial activity of *P. dulce* seed collected from Hail region could be resulted mainly because of the presence multiple fatty acids (e.g., hexadecanoic and 9-octadecenoic acids) or in a combination with the antimicrobial effect of D-turanose sugar.

### 3.2. Antibacterial Activity of *Pithecellobium dulce* Extract

Antimicrobial activity of *P. dulce* extract was assessed against various clinical isolates, including Gram-positive and Gram-negative bacteria. Inhibitory zones (ZOI) and MIC values were determined for each tested bacterial isolate (Table 2). The tested extract has inhibited the growth of the investigated Gram-positive and Gram-negative bacteria with similar potency, although slightly bigger zone of inhibition towards Gram-positive bacteria (*S. aureus*) was observed. MIC values among tested Gram-positive and Gram-negative bacteria towards studied extract are close to each other, which were determined as 233 mg/mL and 300 mg/mL of the extract for *A. baumannii* and *S. aureus*, respectively. It is evident that *P. dulce* seed possesses broad spectrum of activity towards Gram-positive and Gram-negative tested bacterial strains with almost similar MIC values [13]. Current data of the extract showed MBC to MIC ratio of less than 4 times, suggesting that the extract exhibited bactericidal effect. It was reported that *P. dulce* pulp extract possessed similar bactericidal activity [36]. Interestingly, the potent activity of the extract towards drug-resistant *A. baumannii* and other tested drug-resistant clinical strains of *S. aureus* and *E. coli* suggests a completely novel mode of action of the extract. This is because the extract kills *A. baumannii* strain that is resistant to all drugs except colistin as well as inhibiting the growth of drug-resistant *S. aureus* strains. In addition, colistin is well known for its narrow spectrum towards Gram-negative bacteria only [37] indicating that the extract possesses mechanism of action unlike colistin and all other tested inactive drugs making the probability of developing resistance towards this extract very low/limited. This finding would show the importance of this extract as it can be potentially used to treat superbug pathogenic bacteria.

Nevertheless, testing wider range of Gram-positive and Gram-negative bacteria against *P. dulce* seed extract would be of a great value. This will even facilitate in identifying the compound behind the activity based of spectra. This is because similar spectrum of activity was reported for extracts from leaves [30] and roots [16] of *P. dulce* and now for the seed. Similar spectrum of activity with slightly different MIC might be inconclusive as it can be resulted from the overall purity of the active compound and the followed method of extraction. Furthermore, it is very logic to test *P. dulce* extracts against clinical bacterial strains, but including multiple reference strains would be more practical to establish a sensible and rational comparison of spectra among different extracts.

### 3.3. In Silico Simulation and Molecular Interactions

*S. aureus* is a common human pathogen causing various infections ranging from superficial skin infections to severe and life-threatening condition including sepsis, pneumonia, or bone and joint infections [38]. In addition, hospital-acquired infections are well associated with *S. aureus*, and these facts would make this bacterium as good candidate for studying simulation and molecular interactions [39]. Tyrosyl-tRNA synthetase and type IIa topoisomerase that are crucial components for *S. aureus* growth and protein synthesis were then selected and subjected to in silico analysis to predict its molecular interactions with different identified phytochemicals [22]. Various compounds showed negative binding energy with variable potentialities (Table 3), although the highest negative value indicates better energy and docking [40]. This is mainly due to the various 3D chemical structures of tested compounds [24]. In this context, the highest negative energy values were predicted for D-turanose followed by inositol for both 1JIJ and 2XCT macromolecules (Table 3). D-Turanose interaction has resulted in -7.4 and -6.6 kcal/mol for 1JIJ and 2XCT macromolecules, while inositol showed energy values (−7.2 and −5.4 kcal/mol) for the same receptors, respectively (Table 3). This finding indicates efficient interaction of these compounds with targeted receptors, which would mean that one or combination of these compounds is responsible for the inhibition of *S. aureus* growth and explain the antimicrobial activity of the extract (Table 2). Furthermore, conventional hydrogen bounds of 1JIJ-turanose complex was determined as the highest value among all tested complexes (Table 3). Although the highest value of conventional hydrogen bounds through the 2XCT macromolecule was determined for 2XCT-altronic acid complex, 2XCT-turanose showed relatively high value (Table 3). D-Turanose and inositol were predicted to establish hydrogen bonds, which were supported by a network of electrostatic bonds (Figures 1 and 2), and the presence of such bonds is important in the field of pharmacology and drug designing [24]. It was also outlined that the majority of extract compounds interacted with sufficient number of key residues and were deeply embedded in the catalytic regions of both receptors (Table 3). In fact, the distance to the closest interacting residue varied between 1.73 and 2.95 Å.

Altogether, it could be deduced that tyrosyl-tRNA synthetase and type IIa topoisomerase, which inhibit *S. aureus* growth, could be targeted by our identified compounds. In fact, type IIa topoisomerase is considered as major group of both anticancer and antimicrobial drug targets [41]. This was enforced by the interactions of the assessed compounds with tyrosyl-tRNA synthetase (1JIJ). Similar findings were reported by previous reports which outlined significant antibacterial activities based on the occupied areas, molecular interactions, and binding affinities [42]. Moreover, synergistic effect might occur due to the nature of the current extract as containing mixture of phytochemicals [25].

### 3.4. Bioavailability Studies

In silico prediction of bioavailability and drug-likeness properties remains a key criterion in screening drug candidates at the earlier phase of drug discovery and development. They assess the chance for a molecule to become an oral drug with respect to bioavailability aspect in human body [43]. Inositol, hexadecanoic acid, and indole-1-acetic acid predictions were found to obey Lipinski's rule of five which exhibit a total polar surface area (TPSA) less than 122 Å^2^ (Table 4). Physiochemical parameters of the selected compounds reported as been associated with various activities, including antimicrobial, are within the recognized values. They displayed bioavailability score in the range of 55-85%, which are non-P-glycoprotein (P-gp) substrates, hence confirming their high absorption from the gastrointestinal (GI) tract with the exception of D-turanose and inositol which showed low predicted GI absorption (Table 4). Their skin permeation (LogKP) parameters are in the range -11.92 to -2.77, inferring low skin permeability. In major cases, they predicted as noninhibitors of cytochrome P450 isoenzyme (CYP1A2, CYP2C19, CYP2C9, CYP2D6, and CYP3A4) probes. In addition, the bioavailability radar gave a main scan of the drug-likeness of D-turanose, inositol, hexadecanoic acid, and indole-1-acetic acid, (Figure 3), which highlight their predicted oral bioavailability. Nevertheless, although the current study highlighted the potential antibacterial activity of P. dulce seed extract, there are certain limitation and potential directions for further validation and testing. The total yield of each component of the extract detected by the GC may not reflect the actual percentage in the P. dulce seed. For example, detected percentage of fatty acids and esters in the current study was underestimated when compared with similar work conducted on the same seeds. This may be due the real variation among utilised method of extraction, purification, and gas chromatography or their conditions which can lead different experimental yield. It was reported that fatty acids will be underestimated as they do not fly well under the conditions of the current analysis, but performing preliminary separation of the oil would detect percentage of fatty acids accurately [44]. Namely, experimental yield of components detected by GC from one type of plant or its seed is heavily relented on the used methods and/or its conditions.

Although the main focus of the current study is to determine the antibacterial activity, phytochemicals analysis, and in silico interaction of *P. dulce* extract, further essential studies need to be conducted to confirm the antimicrobial activity and evaluate the potential use of the active compound/s in the current extract as therapeutic product treating bacterial infections caused by MDR bacteria in human. Firstly, even the potential antimicrobial activity of proposed compounds (D-turanose and inositol) was previously reported, their in vitro and in vivo activity should be tested against various bacterial isolates including MDR for further confirmation. In addition, results of docking analysis can be confirmed by enzyme biochemical assays. Moreover, other in vivo studies, mode of action, physicochemical properties, toxicity, and resistance testing are all worth conducting for potential active compounds of the extract. Data resulted from these future investigations would confirm the in vitro and in vivo activity of the active compound/s within the current extract and determining its safety status for therapeutic use in human health.

## 4. Conclusions

The current study has investigated phytochemical profiles and antibacterial activity of *Pithecellobium dulce* seed extract (Hail, Saudi Arabia) as well as identifying potential compounds behind the antibacterial activity and their physicochemical, pharmacokinetic, and drug-likeness properties to evaluate its future use to treat infections caused by drug-resistant bacteria in human. The extract inhibited the growth of multiple drug-resistant clinical isolates, including *S aureus*, *E*. *coli*, and *A. baumannii* with similar MIC values. Bioinformatic analysis showed decent interaction of certain compounds (mainly D-turanose and inositol) with tested receptors (tyrosyl-tRNA synthetase and type IIa topoisomerase) of *S. aureus* providing higher probability of being responsible for the antibacterial activity. Furthermore, ADMET analysis revealed desirable bioavailability for tested compounds of the extract indicating its great potential use as antibacterial angsts. This investigation demonstrated *P. dulce* seed as being a rich source for novel antimicrobial agents to treat drug-resistant bacteria potentially by new mode of action and limited/low resistance development. Moreover, the in silico analyses are great tools with short cut for identifying compounds with antimicrobial activity as well as assessing its suitability for the targeted application.

## Figures and Tables

**Figure 1:** 3D illustration (a, b) and the corresponding 2D diagram of interactions for the compounds with the best docking scores, D-turanose (a), and inositol (b) with the active site of 1JIJ. Dotted lines; green and light green: conventional H-bond and carbon hydrogen bond interactions, respectively.

**Figure 2:** 3D illustration (a, b) and the corresponding 2D diagram of interactions for the compounds with the best docking scores, D-turanose (a) and inositol (b) with the active site of 2XCT. Dotted lines; green and grey: conventional H-bond and halogen (manganese, Mn) bond interactions, respectively.

**Figure 3:** Bioavailability radar of the selected compounds including D-turanose, inositol, hexadecanoic acid, and indole-1-acetic acid based on physicochemical indices ideal for oral bioavailability. LIPO: lipophilicity (−0.7 < XLOGP3 < *þ* 5); SIZE: molecular size (175 g/mol < mol.wt.<353 g/mol); POLAR: polarity (20 Å^2^ < (topological polar surface area) TPSA < 130 Å^2^); INSOLU: insolubility (0 < Log S (ESOL) < 6); INSATU: in saturation (0.25 < Fraction Csp3 < 1); FLEX: flexibility (0 < Number of rotatable bonds < 9). The coloured zone is the suitable physicochemical space for oral bioavailability.

**Table 1:** Phytochemical profile of *Pithecellobium dulce* seed extract.

No.	Compound name	Intensity (%)	Retention time (min)	Molecular weight (g/mol)	Chemical formula
1	D-Turanose	55.82	25.97	342.30	C_12_H_22_O_11_
2	Hexadecanoic acid	11.56	20.99	256.42	C_16_H_32_O_2_
3	Indole-1-acetic acid	11.42	22.63	175.18	C_10_H_9_NO_2_
4	Inositol	5.78	19.97	180.16	C_6_H_12_O_6_
5	Octadecanoic acid	4.36	22.8	284.50	C_18_H_36_O_2_
6	Dihydroxyacetone	1.58	26.39	90.08	C_3_H_6_O_3_
7	Methyl heptadecanoate	1.36	19.76	284.50	C_18_H_36_O_2_
8	D-gluco-hexodialdose	0.83	19.06	178.14	C_6_H_10_O_6_
10	Myo-inositol	0.74	21.31	180	C_6_H_12_O_6_
119	Altronic acid	0.65	25	196.16	C_6_H_12_O_7_
10	11-Eicosenoic acid	0.37	24.19	310.50	C_20_H_38_O_2_
11	9-Octadecenoic acid	0.33	26.64	282.50	C_18_H_34_O_2_
12	Methyl elaidate	0.31	21.51	296.50	C_19_H_36_O_2_
13	Hexanoic acid	0.24	8.08	116.16	C_6_H_12_O_2_
14	2-Deoxy-galactopyranose	0.24	28.5	164.16	C_6_H_12_O_5_
15	Ribitol	0.2	19.68	152.15	C_5_H_12_O_5_
16	2-Phenyl-1,2-propanediol	0.17	17.4	152.19	C_9_H_12_O_2_
17	Monomethyl phosphate	0.16	9.66	112.02	CH_5_O_4_P
18	9,10-Dihydrooctadecanoic acid	0.16	23.32	353.40	C_18_H_34_Cl_2_O_2_
19	2,3-Butandiol	0.14	7.4	90.12	C_4_H_10_O_2_
20	D-Mannose	0.14	19.54	180.16	C_6_H_12_O_6_
21	Lyxose	0.12	28	150.13	C_5_H_10_O_5_
22	Azelaic acid	0.11	18.3	188.22	C_9_H_16_O_4_
23	Methyl octadecanoic acid	0.09	25.2	298.50	C_19_H_38_O_2_
24	9,12-Octadecadienoic acid	0.07	21.44	280.40	C_18_H_32_O_2_

**Table 2:** Inhibitory zones (ZOI), minimum inhibitory concentration (MIC), and minimum bactericidal concentration (MBC) of Pithecellobium dulce seed extract towards Gram-positive and Gram-negative clinical bacterial strains.

Bacterial strain	ZOI ceftriaxone (mm)	ZOI extract (mm)	MIC [mg/mL (extract)] ± SD^∗^	MBC [mg/mL(extract)] ± SD^∗^	MBC/MIC ratio
*Methicillin-resistant Staphylococcus aureus [UNI 001]*	14	10	300	600	2
*Staphylococcus aureus [UNI 217]*	16	9	300	600	2
*Staphylococcus aureus [UNI 211]*	27	11	300	600	2
*Staphylococcus aureus [UNI 22]*	30	10	300	600	2
*Escherichia coli [UNI001]*	11	9	300	750	2.5
*Acinetobacter baumannii [UNI002]*	0	9	233 ± 115	600	2.6

Determined minimal inhibitory concentration expressed as the mean of three replicates (mg/mL ± SD). SD: standard deviation ^∗^ zero SD means that three replicates give the same MIC or MBC; mm: millimetre.

**Table 3:** Binding energy, conventional hydrogen bonds, and the closest interacting residues of 1JIJ and 2XCT for TyrRS and gyrase from *S. aureus*, respectively, complexed with the identified compounds.

Compound name	Binding energy (kcal/mol)		Conventional H-bonds		Closest interacting residue (distance, Å)	
	1JIJ	2XCT	1JIJ	2XCT	1JIJ	2XCT
D-Turanose	−7.4	−6.6	10	7	Asp40 (2.01)	Gly584 (1.82)
Hexadecanoic acid	−5.8	−4.0	4	3	Asp 40 (2.29)	Asp1427 (2.38)
Indole-1-acetic acid	−7.1	−5.8	2	3	Gln174 (2.55)	Asp1024 (1.88)
Inositol	−7.2	−5.4	6	8	Tyr170 (1.73)	Arg1012 (2.29)
Octadecanoic acid	−6.0	−5.1	3	1	Asp80 (2.12)	Gln1095 (2.07)
Dihydroxyacetone	−4.1	−3.4	6	4	Gln174 (2.09)	Arg629 (1.98)
Methyl ester of heptadecanoic	−6.2	−4.6	2	1	Lys84 (2.12)	Gly1106 (2.79)
D-Gluco-hexodialdose	−6.3	−4.5	7	7	Asp40 (2.35)	Gly1178 (2.14)
Myo-inositol	−7.2	−5.4	8	6	Asp177 (1.97)	Asp1024 (2.12)
Altronic acid	−6.1	−4.8	8	9	Gln174 (2.04)	Arg601 (1.95)
11-Eicosenoic acid	−6.1	−5.3	2	1	Asn124 (2.29)	Arg1495 (2.54)
9-Octadecenoic acid	−5.0	−4.1	4	6	Gln196 (2.20)	Arg629 (2.18)
Methyl ester of 9-octadecenoic	−6.0	−4.7	5	1	Asp40 (1.99)	Glu1447 (2.19)
Hexanoic acid	−6.1	−5.2	1	1	Gln174 (2.71)	Lys1130 (2.23)
2-Deoxy-galactopyranose	−5.0	−3.7	3	4	Gln190 (2.30)	Ile1289 (1.97)
Ribitol	−6.6	−5.2	7	6	Gln174 (2.21)	Arg629 (2.00)
2-Phenyl-1,2-propanediol	−5.5	−4.2	8	6	Gln174 (2.09)	Asp1024 (2.07)
Monomethyl phosphate	−6.1	−5.2	3	2	Gln174 (1.91)	Asp1142 (1.77)
9,10-Dihydro octadecanoic acid	−4.2	−4.0	5	4	Gln174 (2.13)	Arg1047 (2.18)
2,3-Butandiol	−6.9	−5.2	6	4	Gly193 (2.05)	Asn1269 (2.31)
D-Mannose	−4.4	−3.5	6	5	Gln196 (2.19)	Lys446 (2.17)
Lyxose	−6.6	−5.5	5	9	Gln190 (1.95)	Arg517 (1.85)
Azelaic acid	−6.1	−4.6	5	6	Asp40 (2.24)	Thr507 (1.93)
Methyl ester of octadecanoic acid	−6.2	−4.4	6	6	Gln174 (2.17)	Arg1092 (2.12)
9,12-Octadecadienoic acid	−6.0	−5.2	2	1	Gly193 (2.14)	Lys1373 (2.95)

**Table 4:** Pharmacokinetics properties of the selected compounds of the extract.

Compounds	D-turanose	Inositol	Hexadecanoic acid	Indole-1-acetic acid
Physicochemical properties/lipophilicity/drug-likeness				
Molecular weight (g/mol)	342.30	180.16	256.42	175.18
Num. heavy atoms	23	12	18	13
Num. arom. heavy atoms	0	0	0	9
Fraction Csp3	1.00	1.00	0.94	0.10
Num. rotatable bonds	4	0	14	2
Num. H-bond acceptors	11	6	2	2
Num. H-bond donors	8	6	1	1
Molar refractivity	68.16	35.81	80.80	49.78
TPSA	189	121.38	37.30	42.23
Lipinski's rule	No	Yes	Yes	Yes
Bioavailability score	0.17	0.55	0.85	0.85
Bioavailability				
GI absorption	Low	Low	High	High
BBB permeability	No	No	Yes	Yes
P-gp substrate	Yes	Yes	No	No
CYP1A2 inhibitor	No	No	Yes	Yes
CYP2C19 inhibitor	No	No	No	No
CYP2C9 inhibitor	No	No	Yes	No
CYP2D6 inhibitor	No	No	No	No
CYP3A4 inhibitor	No	No	No	No
LogKp (cm/s)	-11.92	-10.03	-2.77	-5.62

## Data Availability

All data that support the findings of this study are available within the article.
